The article "Expression and Role of TRIM2 in Human Diseases" was published in 2022. Journal: Biomed Res Int.

# Expression and Role of TRIM2 in Human Diseases

**DOI:** 10.1155/2022/9430509

**Published:** 2022-08-23

**Authors:** Maolin Xiao, Jianjun Li, Qingyuan Liu, Xiangbiao He, Zongke Yang, Delin Wang

**Affiliations:** ^1^Department of Urology, Chongqing General Hospital, No. 118, Xingguang Avenue, Liangjiang New Area, Chongqing 401147, China; ^2^Department of Urology, The First Affiliated Hospital of Chongqing Medical University, No. 1 Youyi Road, Yuanjiagang, Yuzhong District, Chongqing 400016, China; ^3^Department of Spinal Surgery, Zhujiang Hospital, Southern Medical University, No. 253, Industrial Avenue Middle, Haizhu District, Guangzhou, Guangdong 510000, China; ^4^Department of Urology, Dianjiang People's Hospital of Chongqing, No. 116 North Street, Guixi Street, Dianjiang, Chongqing 408399, China

## Abstract

Tripartite motif (TRIM) protein family proteins contain more than 80 members in humans, and most of these proteins exhibit E3 ubiquitin ligase activity mediated through a RING finger domain. Their biological functions are very complex, and they perform diverse functions in cell evolution processes, such as intracellular signaling, development, apoptosis, protein quality control, innate immunity, autophagy, and carcinogenesis. Tripartite motif-containing protein 2 (TRIM2), a member of the TRIM superfamily, is an 81 kDa multidomain protein, also known as CMT2R or RNF86, located at 4q31.3. TRIM2 functions as an E3 ubiquitin ligase. Current studies have shown that TRIM2 can play roles in neuroprotection, neuronal rapid ischemic tolerance, antiviral responses, neurological diseases, etc. Moreover, based on some studies in tumors, TRIM2 regulates tumor proliferation, migration, invasion, apoptosis, and drug resistance through different mechanisms and plays a critical role in tumor occurrence and development. This review is aimed at providing a systematic and comprehensive summary of research on TRIM2 and at exploring the potential role of TRIM2 as a biomarker and therapeutic target in many kinds of human diseases.

## 1. Introduction

Tripartite motif (TRIM) proteins constitute a medium-sized subfamily mainly consisting of posttranslational modifiers. The TRIM family has more than 80 members [1], and the genomes of most eukaryotes encode TRIM proteins. The total number of TRIM genes is related to the level of biological evolution. For example, there are over 70 TRIM family members in humans, approximately 64 in mice, 20 in worms, and approximately 10 in flies, indicating extensive evolution [2, 3]. TRIM proteins regulate multiple biological processes, and their functions range from antiviral defense and regulation of immune and cellular stress responses to the regulation of cell proliferation, apoptosis, cell differentiation, transcription, and DNA repair [3, 4].

The TRIM is always located towards the N-terminus of the protein and the order of, as well as the spacing between individual these domains, is highly conserved; TRIM proteins contain three types of domains, namely, a RING finger domain, one or two B-box-type zinc finger (BB1 and BB2) domains, and a coiled-coil (CC) domain [2, 5]. The RING domain constitutes the catalytic center of TRIMs and confers E3 ligase activity; TRIM proteins can thus ubiquitinate substrates as components of the ubiquitin–proteasome system [6, 7]. However, not all TRIM proteins have a RING finger domain: eight of the TRIM proteins in humans are RING-less TRIM proteins [2]. The B-box and CC domains mediate protein–protein interactions, and previous studies have proposed that the B-box domain, together with the CC domain, provides binding sites for ubiquitinated substrates through the RING domain [8, 9].

The carboxyl terminal (C-terminal) domains are different as indicated by the overall domain structure and distinct C-terminal domains of TRIMs and can be classified into several subgroups [10]. These domains include the COS domain, fibronectin type III repeat (FNIII), PRY domain, SPRY domain, acid-rich region (ACID), filamin-type IG domain (FIL), NCL-1, HT2A, and Lin-41 (NHL) domain, PHD domain, bromodomain (BROMO), meprin and TRAF-homology domain (MATH), ADP-ribosylation factor family domain (ARF), and transmembrane region (TM) [2].

Tripartite motif-containing protein 2 (TRIM2) is an 81 kDa multidomain protein, also known as CMT2R or RNF86, located at 4q31.3. TRIM2 belongs to subgroup VII, whose members contain FIL domains and NHL repeats at their C-termini [11] (Figures 1(a) and 1(b)). Only 4 mammalian TRIM proteins belong to this subgroup: TRIM2, TRIM3, TRIM32, and TRIM71 [11–13]. The RING domain of TRIM2 has been found to mediate ERK-dependent ubiquitination of BCL-2-interacting mediator of cell death (Bim). After phosphorylation by ERK, TRIM2 binds to phosphorylated Bim and mediates its degradation [14]. The filamin domain, together with the CC domain, was proposed to recruit proteins regulating mRNA translation [15]. NHL repeats are generally considered to be structural units involved in protein binding [16].

In the initial study of TRIM2, TRIM2 was shown to be mainly expressed and play a role in the brain. TRIM2 was first related to neuroplasticity of the minor muscle, where it interacts with myosin V through its NHL domain [17]. TRIM2 plays an important role in both malignant and nonmalignant diseases. This review focuses on TRIM2-related research and development in various fields, including both nonmalignant diseases and cancers.

## 2. The Functions of TRIM2 in Nonmalignant Diseases

### 2.1. TRIM2 in Neurogenesis, Development, and Neuronal and Axonal Differentiation

Changes in TRIM2 expression have long been related to human nervous system diseases, and TRIM2 plays an important role in the nervous system [18]. Using a bioinformatics database, Su et al. found that TRIM2 is an important gene that participates mainly in the regulation of the cell component tissue, axonogenesis, and cell morphogenesis during neuronal differentiation and is regulated by the upstream microRNAs (miRNAs) hsa-miR-18a-5p, hsa-miR-181b-5p, and hsa-miR-181d-5p [19]. Previous studies have confirmed that TRIM2 inhibits the expression of Bim during rapid ischemic tolerance in the nervous system and then regulates p42/p44 MAPK-dependent ubiquitination, thus playing a neuroprotective role [14].

Balastik et al. found that TRIM2 binds to neurofilament light subunit (NF-L) and regulates its ubiquitination; furthermore, they showed that TRIM2-deficient mice exhibit accumulation of NF-L in neuronal structures, which leads to axonal diseases, progressive neurodegeneration, tremors, and the onset of ataxia at a young age [20]. In another study, Khazaei et al. sought to determine whether TRIM2 regulates the NF-L level in hippocampal neurons and found that NF-L immunoreactivity was greatly reduced after TRIM2 overexpression, while the level of NF-L was significantly increased after TRIM2 knockdown. To further investigate whether NF-L is indeed a downstream ubiquitination target of TRIM2, they coexpressed NF-L with either wild-type TRIM2 or a TRIM2 mutant lacking the ubiquitin ligase domain (TRIM2*Δ*RBCC) [20] in 293T cells and analyzed NF-L levels and ubiquitination. TRIM2 mediates the polyubiquitination of NF-L and thereby reduces the NF-L level, while the ubiquitin ligase-deficient TRIM2 mutant could not reduce the level of NF-L; thus, TRIM2 may be a key regulator of axonal outgrowth [21]. Moreover, as a downstream target of miR-181c, TRIM2 expression can be inhibited by miR-181c, an event closely related to the development of progressive neurodegeneration with juvenile tremor and ataxia [22].

Recently, TRIM2 has been shown to act as a cofactor to confer substrate specificity in the interaction between the ubiquitin ligase neural precursor cell-expressed developmentally downregulated gene 4 (NEDD4-1) and two ATP-binding cassette (ABC) transporters involved in cholesterol homeostasis [23]. These findings suggest that TRIM2 is a key regulator of neuronal differentiation.

Beyond the key role of TRIM2 in neuronal growth and regulation, Lokapally et al. found in a study in Xenopus that TRIM2 was related to programmed cell death 6-interacting protein/apoptosis-related gene-2-interacting protein X (Pdcd6ip/Alix), which regulates nerve formation and development, controls cell proliferation and cell survival during early neural development, and participates in the determination and differentiation of neural progenitors; these findings provide evidence for a TRIM2-Alix interaction during early neural development [18].

### 2.2. TRIM2 in Charcot-Marie-Tooth Disease (CMT)

CMT is a clinically and genetically heterogeneous polyneuropathy (distal symmetric polyneuropathy (DSP)) characterized by progressive and length-dependent degeneration of peripheral nerves and resulting in muscle weakness and emaciation of distal limbs, progressive foot deformities, walking disorders, and sensory deficiencies. The age of onset and clinical severity are highly variable [24]. Based on neurophysiological and pathophysiological criteria, CMT is divided into two main types: demyelinating and axonal. CMT type 2 (CMT2) belongs to the axonal type, which is characterized by distal muscle weakness and atrophy, mild sensory loss, and normal or near-normal nerve conduction velocities [25]. TRIM2 loss-of-function mutation has been reported to be a rare cause of the autosomal recessive disease CMT type 2 (CMT2R; OMIM 615490), causing neurofilament accumulation and axon degeneration both in patients and in a mouse model [26, 27]. A compound heterozygous mutation in the TRIM2 gene was found in a patient with early-onset neuropathy, and abnormal accumulation of axonal neurofilaments caused by a lack of ubiquitin in TRIM2 may be the potential mechanism of its pathogenesis [26]. Subsequent exon sequencing of a patient with early onset of CMT and bilateral vocal cord paralysis revealed a homozygous TRIM2 mutation; this mutation was embedded in an 18 Mb homozygous region, which may lead to vocal cord paralysis [28]. In a recent study, Magri et al. reported two cases with corresponding clinical manifestations due to TRIM2 mutations. In addition to vocal cord paralysis, the patients manifested other clinical features secondary to several other cranial neuropathies, such as facial muscle weakness, dysphagia, dyspnea, and hearing disorders. Genetic analysis revealed two novel TRIM2 mutations in each patient. This report expanded the genotypic and phenotypic spectrum of TRIM2 deficiency and confirmed that extensive cranial nerve involvement is the core feature of the CMT2 subtype, which provided a foundation for further study of the disease [29].

### 2.3. TRIM2 in Glaucoma

In a study on the effect of miR-145-5p on apoptosis in retinal ganglion cells (RGCs) in glaucoma, the researchers established a rat glaucoma model and found that silencing miR-145-5p improved glaucoma symptoms, promoted the survival of RGCs, and inhibited their apoptosis *in vitro*. After overexpression of miR-145-5p, only TRIM2 was significantly downregulated. In RGCs treated with N-methyl D-aspartic acid (NMDA), both the mRNA and protein expression of TRIM2 was decreased. Finally, a luciferase reporter assay confirmed that TRIM2 is the downstream target of miR-145-5p. A series of functional experiments have indicated that upregulation of TRIM2 can inhibit RGC apoptosis *in vitro*. Further studies on possible pathways regulated by TRIM2 showed that the levels of phosphorylated PI3K/AKT in RGCs were decreased after NMDA treatment and restored after TRIM2 overexpression; in addition, treatment with LY294002 (30 *μ*m), an antagonist of the PI3K/AKT pathway, reversed the promoting effect of TRIM2 on PI3K/AKT pathway activation. Therefore, TRIM2 promotes RGC activity and inhibits RGC apoptosis through the PI3K/AKT signaling pathway [30].

### 2.4. TRIM2 in Antiviral Infections

In earlier studies, TRIM2 was found through a yeast two-hybrid screen to bind to signal regulatory protein *α* (SIRPA/SHPS1) [31]. SIRPA is a modulator of phagocytosis [32] that, similar to TRIM2, is expressed in both myeloid and neuronal cells [33] and also in macrophages [34]. In a relevant research, TRIM2 was found through *in vivo* experiments in mice to play a unique antiviral role by interacting with SIRPA to block cellular entry of hemorrhagic fever New World arenavirus (NWA). In *in vitro* and *in vivo* studies, the binding of phosphorylated SIRPA to TRIM2 was verified by reverse transcription–polymerase chain reaction (RT–PCR) to block virus internalization, and at least the FIL domain but not the RING domain, which encodes ubiquitin ligase activity, was found to be required for the antiviral activity of TRIM2. In addition, the researchers analyzed relative phagocytosis by incubating bone marrow-derived macrophages (BMDMs) isolated from TRIM2 knockout and wild-type mice with phrodo Red-labeled apoptotic thymocytes and found that loss of TRIM2 led to increased macrophage engulfment of apoptotic cells, a process known to be regulated by SIRPA [35, 36]. These findings suggested the presence of overlap among the pathways mediating NWA entry and phagocytosis and may contribute to a better understanding of the role of TRIM2 in macrophage and neuronal cell function in addition to its role in virus entry [37].

In another study, researchers explored changes in TRIM gene expression in normal human dermal fibroblasts (NHDFs) with and without lipopolysaccharide stimulation during porcine endogenous retrovirus (PERV) infection. The expression profile of TRIMs was evaluated by oligonucleotide microarray analysis and RT–PCR. Nine genes (TRIM1, TRIM2, TRIM5, TRIM14, TRIM16, TRIM18, TRIM22, TRIM27, and TRIM31) were significantly differentially expressed, among which the expression of TRIM2 was increased; however, the mechanism needs further study [38, 39]. The results of these studies may provide a better understanding of the antiviral role of TRIM2.

### 2.5. TRIM2 in Angiogenesis

A study by Wong et al. confirmed that among the genes studied in conditional angiogenesis, TRIM2 was significantly upregulated under hypoxic and inflammatory conditions, which in turn promoted angiogenesis; the mechanism may be related to recombinant high-density lipoprotein (rHDL). Under hypoxic and inflammatory conditions, TRIM2 knockdown by lentiviral transduction impaired the development of fibroblasts and weakened the angiogenic effect of rHDL. In addition, TRIM2 knockdown weakened the ability of rHDL to increase renal tubule formation under hypoxia. This research suggests that TRIM2 may be a new regulator of rHDL that promotes angiogenesis during hypoxia [40].

## 3. The Functions of TRIM2 in Cancers

### 3.1. TRIM2 in Ovarian Cancer

Ovarian cancer is one of the most common reproductive malignancies and has the highest mortality rate among all gynecological malignancies. Approximately 70% of patients have advanced-stage disease at diagnosis [41, 42].

p85*β* is an oncogenic factor that promotes tumorigenesis and tumor progression [43]. A study indicated that p85*β* alters the response of ovarian cancer to EGFR inhibitors through p38 MAPK-mediated regulation of DNA repair [44]. The receptor tyrosine kinase AXL is overexpressed in multiple cancer types, including ovarian cancer, causing malignant phenotypes and a poor prognosis [45–47]. In a study on ovarian cancer progression, high TRIM2 expression was found to promote the proliferation and invasion of ovarian cancer cells. In addition, P85*β* regulates the autophagic degradation of AXL, which leads to activation of oncogenic signaling, and TRIM2 is the E3 ligase for AXL. The mechanism may be related to the p85*β*-induced change in the phosphorylation level of TRIM2, which mediates the selective regulation of AXL by p85*β*, disrupts autophagic degradation of the AXL protein, and regulates the occurrence and development of tumors [48]. In another study, related gene sequencing experiments confirmed that the expression of miR-145 in ovarian cancer tissues and cell lines was consistently downregulated compared with that in normal ovarian tissues and further confirmed that TRIM2 was the downstream target gene of miR-145. The direct relationship between miR-145 and TRIM2 was confirmed by a dual luciferase reporter assay. In a further mechanistic study, according to Thompson et al. [14], TRIM2 mediated ERK-dependent ubiquitination of Bim in other cell types, TRIM2 was downregulated after transfection with miR-145, and Bim was upregulated in ovarian cancer cells. Under baseline conditions, TRIM2 showed diffuse cytoplasmic staining, consistent with its role as an E3 ubiquitin ligase [49].

### 3.2. TRIM2 in Cervical Cancer

Cervical cancer is the second leading cause of death among gynecological malignancies, and most confirmed cases are in developing countries, where screening and prevention efforts are limited. In the United States, 4290 patients died of cervical cancer in 2020 [50].

In a study to screen for differentially expressed genes in cervical cancer, two groups of cervical squamous cell carcinoma (SCC) tissues and adjacent normal squamous epithelium were subjected to cDNA microarray analysis. The TRIM2, S100A2, GPC4, p72, IGFBP-5, and NAB2 genes were selected and evaluated by RT–PCR. No consistent difference in the mRNA expression level of any of these genes except IGFBP-5 was found between cancer tissue and normal cervical squamous epithelium. The expression of TRIM2 in tumor tissue was slightly lower than that in adjacent tissue, but the difference was nonsignificant [51]. Due to the comparative lack of research findings, either TRIM2 does not play a role in cervical cancer or whether it plays a role needs further verification *in vivo* and *in vitro.*

### 3.3. TRIM2 in Osteosarcoma

Osteosarcoma is the most common primary malignant bone tumor. Its origin cells produce bone or osteoid as well as different amounts of cartilage matrix and fibrous tissue, which is most common in the metaphysis of long tubular bone [52, 53]. The incidence rate of osteosarcoma is approximately 2-4 cases per million per year, and the morbidity is higher in males than in females [54].

A study on osteosarcoma indicated that TRIM2 may affect the proliferation, migration, and invasion of osteosarcoma cells through the PI3K/AKT signaling pathway and that high TRIM2 expression is associated with a low survival rate and promotion of metastasis. To further verify the regulatory role of TRIM2 at the molecular level, two groups of cell lines with significantly differential gene expression were identified by transcriptome sequencing, and seven differentially expressed genes related to TRIM2 (DDIT3, CREB5, SIRT4, GPR65, FZD8, SHC2, and ART5) were extracted from the expression profile and subjected to Gene Ontology (GO) and Kyoto Encyclopedia of Genes and Genomes (KEGG) pathway enrichment analyses. After silencing TRIM2, all of these genes except for FZD8 and SHC2 were significantly upregulated in both cell lines, as shown by RT–PCR; therefore, it is speculated that TRIM2 can function by regulating five genes that are significantly upregulated in osteosarcoma. The potential downstream target gene of TRIM2 predicted by KEGG pathway enrichment analysis was verified by western blot analysis. After TRIM2 inhibition in osteosarcoma cell lines, the protein level of p-AKT was decreased, while the level of AKT showed no significant change. In addition, the protein levels of PKA, CREB, and p-CREB were not affected upon TRIM2 inhibition in osteosarcoma cell lines, suggesting that TRIM2 regulates the progression and metastasis of osteosarcoma through the PI3K/AKT signaling pathway [55].

### 3.4. TRIM2 in Neuroblastoma

Neuroblastoma (NB) is a common extracranial tumor in children, accounting for 15% of childhood cancer deaths and threatening the lives and health of children worldwide [56]. Approximately 700 cases are diagnosed annually in the United States alone [57].

Salmena et al. first proposed the competitive endogenous RNA (ceRNA) hypothesis [58]. As a downstream target, TRIM2 is also regulated by upstream long noncoding RNAs (lncRNAs) and miRNAs. As shown in some studies, the lncRNA NR2F1-AS1 could act as an oncogene in malignant tumors such as osteosarcoma and endometrial carcinoma [59, 60]. miR-493 could target downstream genes to inhibit tumor proliferation [61, 62]. Upregulation of TRIM2 expression has recently been shown to promote the growth of neuroblastoma cells. Moreover, researchers found that NR2F1-AS1 was highly expressed in neuroblastoma tissues and that its knockdown inhibited the proliferation and invasion of tumor cells. After silencing of miR-493, the effect of NR2F1-AS1 on tumor cells was reversed. As a downstream target gene, TRIM2 regulates the occurrence and development of neuroblastoma in cooperation with its upstream mediators, and the relationship between TRIM2 and miR-145 was verified by a dual luciferase reporter assay. The NR2F1-AS1/miR-493 axis was concluded to promote the progression of neuroblastoma by regulating TRIM2 [63].

### 3.5. TRIM2 in Breast Cancer

Breast cancer is heterogeneous cancer and has the highest incidence and the second highest mortality in women among all cancers [64]. Because three-quarters of breast cancer patients are positive for hormone receptor (HR) expression, tamoxifen (TAM) remains an important treatment option for luminal breast cancer patients and a first-line treatment for premenopausal patients [65, 66].

The protein SRY-related high-mobility-group box 10 (Sox10) is a member of the Sox transcription factor family, whose members are involved in the development of neural crest cells [67]. Recently, higher expression of Sox10 was reported to be significantly associated with high-grade tumors, late-stage tumors, and tumors with metastatic involvement of four or more lymph nodes [68]. To date, there have been few functional experiments investigating the relationship between TRIM2 and breast cancer. Panaccione et al. identified the characteristics of the SOX10/PROM1 gene through bioinformatics analysis. The expression of TRIM2 in basal-like breast carcinoma (BBC) is related to that of SOX10, and the expression of TRIM2 in breast cancer is clearly abnormal. This finding provides new ideas for further basic research, diagnosis, prognosis prediction, and clinical research [69].

In a study of tamoxifen resistance, TRIM2 was found to be highly expressed in the TAM-resistant breast cancer cell line MCF-7R, while the expression of Bim was significantly decreased. The binding of TRIM2 to Bim in MCF-7R cells was confirmed by coimmunoprecipitation assays. Further experiments showed that the TRIM2 protein level was regulated by the GPER-MAPK/ERK signaling pathway and that activation of the GPER-MAPK/ERK signaling pathway led to an increase in the TRIM protein level. GPER-MAPK/ERK pathway activation also affected the interaction of TRIM2 and Bim, leading to ubiquitination-mediated degradation of Bim, which plays a key role in the apoptosis of tamoxifen-resistant breast cancer cells [70].

### 3.6. TRIM2 in Follicular Thyroid Carcinoma

Follicular thyroid carcinoma (FTC) is a malignant tumor of the thyroid follicular epithelium that easily invades the capsule and blood vessels [71]. FTC is the most common histological type of epithelial thyroid carcinoma after papillary thyroid carcinoma (PTC) [72, 73] and accounts for 6-10% of all thyroid cancers [74].

TRIM2 is abnormally expressed in thyroid follicular carcinoma. Using the Affymetrix microarray platform (HG-U133A), Williams et al. identified differentially expressed genes in a series of FTCs and indolent tumors with metastatic and invasive biological behavior and conducted long-term follow-up. The differentially expressed genes between invasive FTC and noninvasive FTC were compared. TRIM2 was one of the four differentially expressed genes between the two groups, and its expression in noninvasive FTC was higher than that in invasive FTC [75].

The higher expression of TRIM2 in noninvasive FTC can help to improve the accuracy of FTC diagnosis and play a positive role in treatment and prognostic evaluation. However, the functional expression of TRIM2 and the underlying mechanism in malignant thyroid tumors need further investigation.

### 3.7. TRIM2 in Pancreatic Cancer

The most common type of pancreatic cancer is pancreatic ductal adenocarcinoma (PDAC). Approximately 60,000 new PDAC cases are diagnosed each year, and approximately 50% of patients are diagnosed at an advanced stage [76]. Pancreatic cancer is the seventh leading cause of cancer-related death worldwide, responsible for more than 430,000 related deaths annually [77].

Research on the relationship between TRIM2 and pancreatic cancer revealed that the expression of TRIM2 in pancreatic cancer is significantly increased, which was negatively correlated with the prognosis of pancreatic cancer. TRIM2 silencing can significantly inhibit the proliferation, migration, invasion, and tumorigenicity of pancreatic cancer cells [78]. The increased levels of reactive oxygen species (ROS) in pancreatic cancer cells mediate various tumor-promoting activities [79]. In a subsequent study, the results of RNA sequencing suggested that the downstream differentially expressed genes after TRIM2 silencing were significantly enriched in the “oxidative phosphorylation” and “reactive oxygen species” pathways. The level of ROS in pancreatic cancer cells was significantly decreased by TRIM2 knockdown, and the mechanism may involve the positive correlation of TRIM2 expression with NRF2 expression. Overexpression of TRIM2 reversed the decrease in the ROS level caused by N-acetyl-L-cysteine (NAC). In a further mechanistic study, it was concluded that TRIM2 can accelerate the progression of pancreatic cancer through the ROS-related NRF2/ITGB7/FAK axis, which reveals a new regulatory role of TRIM2 through the regulation of redox homeostasis and integration of independent signaling pathways. The study also confirmed that the expression of p27 (the G1 checkpoint CDK inhibitor) can be increased by TRIM2 knockdown [78]. TRIM2 may thus be a promising biomarker and therapeutic target in pancreatic cancer.

### 3.8. TRIM2 in Melanoma

Melanoma is a cutaneous malignancy caused by malignant transformation of epidermal melanocytes. Its morbidity and mortality have recently increased significantly [80, 81]. Current studies have shown that somatic genetic alterations are associated with melanoma and that the BRAF/RAS/RAF/MEK/ERK signaling pathway is often dysregulated in melanoma [82].

Xia et al. studied the role of the TRIM family in the prognosis of melanoma through analysis of Oncomine, UCSC Genome Browser, and other related databases. TRIM2 was found to be highly expressed in melanoma, and this finding was verified by qRT–PCR, indicating that TRIM2 plays an important role in the occurrence and development of melanoma. Furthermore, the GEPIA database was used to analyze the prognostic value of TRIM2 in melanoma. Neither high nor low TRIM2 expression had a significant effect on overall survival (OS) and disease-free survival (DFS) [83]. However, the oncogenic role of TRIM2 in melanoma needs to be confirmed by further experiments *in vivo* and *in vitro*, and the oncogenic mechanism remains unclear. In addition, whether TRIM2 is related to the abovementioned pathways needs further exploration.

### 3.9. TRIM2 in Lung Adenocarcinoma

Adenocarcinoma is the most common histological subtype of primary lung cancer, accounting for more than 40% of lung cancer cases [84, 85]. Nintedanib combined with docetaxel has been approved by the European Drug Administration (EMA) as a second-line treatment option for patients with lung adenocarcinoma [86]. Gefitinib is an epidermal growth factor receptor tyrosine kinase inhibitor (EGFR-TKI). Compared with platinum-based chemotherapy, EGFR-TKIs can significantly prolong progression-free survival (PFS) in patients with advanced non-small-cell lung cancer [87].

TRIM2 is highly expressed in lung adenocarcinoma, as measured by qRT–PCR and western blot analysis. In an *in vitro* experiment, the proliferation, colony formation, migration, and invasion of lung adenocarcinoma cells were found to be significantly enhanced after TRIM2 overexpression. In contrast, after TRIM2 knockdown, the opposite effects were observed. Three commonly used molecular drugs including docetaxel, doxorubicin, and gefitinib are used to investigate the effect of TRIM2 expression on the therapeutic sensitivity of lung adenocarcinoma cells. After TRIM2 overexpression and treatment with the three different drugs, the survival rate of TRIM2-overexpressing cancer cells was significantly increased, while the survival rate of TRIM2 knockdown cancer cells was significantly reduced. In addition, analysis of stem cells in pellet culture showed that TRIM2 overexpression effectively promoted the expression of stem cell-related biomarker proteins and mRNAs, such as Bmil, ALDH1, and CD133, indicating that TRIM2 expression was closely related to the sphere-forming ability of tumor stem cells. In further studies, Snail1 was shown to directly interact with TRIM2 in cells. TRIM2 could enhance the proliferation, invasion, and migration of lung adenocarcinoma cells by regulating the ubiquitination-mediated degradation of Snail1. Notably, Snail1 is a marker of epithelial–mesenchymal transition (EMT), revealing that TRIM2 and Snail can regulate EMT in lung adenocarcinoma [88]. Research on TRIM2 can provide more detailed information for further studies on lung adenocarcinoma, including the search for biological targets.

### 3.10. TRIM2 in Colorectal Cancer

Colorectal cancer (CRC) is the third most common cancer diagnosed in men and the second in women, with more than 1.8 million new cases and approximately 861,000 deaths reported in 2018 [89].

Immunohistochemical analysis showed that TRIM2 was highly expressed in tumor tissues in a study of TRIM2 in CRC that also included *in vitro* cell proliferation assays, cell adhesion assays, and Transwell migration and invasion assays. The proliferation, migration, and invasion abilities of CRC cells were significantly enhanced after TRIM2 overexpression, while the cell migration and invasion abilities were decreased after TRIM2 silencing, and the same findings were obtained *in vivo*. Moreover, the expression of TRIM2 was significantly correlated with tumor stage and age but not with sex, body weight, tumor size, tumor differentiation, or preoperative CEA level. The level of TRIM2 in recurrent metastatic tumors was much higher than that in recurrent nonmetastatic tumors. In further mechanistic studies, the expression of TRIM2 was found to be negatively correlated with that of yes-related protein (YAP), and TRIM2 was found to regulate the metastasis of CRC cells through EMT *in vivo* and *in vitro* [90].

### 3.11. TRIM2 in Clear Cell Renal Cell Carcinoma

Approximately 400,000 new cases of renal cell carcinoma were estimated to be diagnosed worldwide in 2018; most of these cases were in patients over the age of 60, and approximately two-thirds were in men [41]. The vast majority of renal cell carcinomas are clear cell renal cell carcinomas (ccRCCs) [91].

Xiao et al. showed that the expression of TRIM2 in ccRCC was significantly lower than that in normal renal tissue by bioinformatics analysis. The Cancer Genome Atlas (TCGA) data analysis showed that TRIM2 expression in T3 and T4 tumors was significantly lower than that in T1 and T2 tumors; moreover, TRIM2 expression in T4 tumors was significantly lower than that in T3 tumors. These results suggested that the expression level of TRIM2 is correlated with TNM stage but not with sex, age, or lymph node metastasis status. Further statistical analysis of the TCGA-kidney renal clear cell carcinoma (KIRC) dataset showed that TRIM2 expression was significantly correlated with tumor recurrence, OS, and DFS. Through gene set enrichment analysis (GSEA), lower TRIM2 expression was found to be associated with the G2/M checkpoint, EMT, hypoxia pathway, and Myc signaling gene sets, and TRIM2 was speculated to possibly play a negative role in regulating cell cycle progression, EMT, and Myc signaling pathways in ccRCC. In an *in vitro* experiment, both the mRNA and protein expressions of TRIM2 in ccRCC cells were significantly lower than those in normal renal epithelial cells and the corresponding noncancerous renal tissues, as determined by qRT–PCR and immunohistochemistry (IHC). TRIM2 overexpression significantly inhibited the migration, invasion, and proliferation of cancer cells [92].

Bioinformatics analysis was used to construct a circRNA-miRNA–mRNA network, and according to the model, TRIM2 was confirmed to be an independent prognostic factor for survival in ccRCC patients. The hsa_circ_0002286/hsa-miR-222-5p/TRIM2 axis was found to play a critical role in the progression of ccRCC. TRIM2 overexpression may inhibit the metastasis and progression of ccRCC. However, no relevant *in vivo* and *in vitro* experiments have been conducted to verify these observations, and further research on the regulation of the ceRNA network in ccRCC is needed [93].

### 3.12. TRIM2 in Oral Buccal Mucosa Cancer

Oral cancer is the fifth most common cancer worldwide and has the highest morbidity and mortality in developing countries. Annually, nearly 300,000 new cases of oral cancer are diagnosed worldwide, and oral cancer results in 145,000 deaths [94]. Known risk factors include smoking, alcoholism, and chewing of betel quid (pan/paan) [95].

TRIM2 was found to be consistently expressed at low levels in buccal mucosa cancer. Yang et al. identified the pathogenic genes related to the occurrence and development of oral buccal mucosa cancer by a whole-genome microarray screen. The golden hamster model of buccal mucosa cancer was established by induction with 9,10-dimethylene-1,2-benzanthracene (DMBA). Venn diagram analysis was performed to identify genes with consistently abnormal expression, and TRIM2 was found to be consistently abnormally expressed in various stages of oral buccal mucosa cancer, which showed consistently low expression; these findings may provide insights for the treatment and chemoprevention of buccal mucosa cancer. However, no relevant *in vivo* and *in vitro* experimental studies have been conducted [96], and it is necessary to further confirm the role of TRIM2 in the occurrence and development of buccal mucosa cancer and to explore the related mechanism.

## 4. Discussion

The above summarized points indicate that TRIM2 plays an important role in several diseases. We summarized the literature in nononcological research, as described above, concentrating mainly on the following aspects: (1) TRIM2 is regulated by the upstream miRNAs hsa-miR-18a-5p, hsa-miR-181b-5p, hsa-miR-181d-5p, and miR-181c and is associated with Pdcd6ip/Alix. In addition, TRIM2 plays a role in neuronal differentiation, axonal growth, and related nervous system diseases [18–21]. (2) TRIM2 inhibits Bim expression during rapid ischemic tolerance in the nervous system and then exerts a neuroprotective effect by regulating p42/p44MAPK-dependent ubiquitination [14, 22]. (3) TRIM2 is the downstream target of miR-145-5p, promotes RGC activity, and inhibits RGC apoptosis through the PI3K/AKT signaling pathway [30]. (4) TRIM2 interacts with SIRPA to block the cellular entry of hemorrhagic fever NWA, indicating that it can play a role in antiviral activity [37] (Figure 2).

The above studies show that TRIM2 can promote angiogenesis and that the mechanism may be related to recombinant rHDL, but the pathway involved in tumor angiogenesis is very complex [97]. Angiogenesis is a process through which new capillaries are formed from preexisting blood vessels and is very important for the growth and metastasis of many solid tumors, including pancreatic tumors [98]. When proangiogenic molecules predominate over antiangiogenic molecules, angiogenesis is activated [99]. To understand the role of TRIM2 in promoting angiogenesis, it is necessary to further investigate whether TRIM2 plays an important role in tumors, either by acting as a cancer-regulating factor or by promoting tumor angiogenesis. In addition, whether TRIM2 can be a biological target for targeted treatment of abnormal tumor angiogenesis and whether any potential signaling pathways related to TRIM2 could be exploited for this purpose must be investigated.

Studies related to TRIM2 in tumors have primarily revealed that it plays a role in promoting tumor growth by fostering tumor proliferation, invasion, and migration, as shown in cancers such as neuroblastoma and pancreatic cancer [63, 78]. Some studies have suggested that TRIM2 is related to tumor stage and patient age. However, in other studies, including studies in ccRCC, FTC, and oral buccal mucosa cancer, TRIM2 has been shown to act as a tumor suppressor [75, 92, 93, 96]. Notably, in a study of cervical cancer, no consistent difference in the expression of TRIM2 was found between cancer tissues and normal cervical squamous epithelium [51] (Table 1). We analyzed the differential expression of TRIM2 in tumor tissues and normal tissues of different organs based on the TCGA and Genotype-Tissue Expression (GTEx) databases, and the results are shown in Figure 3.

In oncological research, we summarized the following findings about TRIM2-related proteins, signaling pathways, or upstream genes based on the available literature: (1) TRIM2 interacts with Bim to regulate tumor progression [49, 70]; (2) TRIM2 regulates tumor progression through the PI3K/AKT, GPER-MAPK/ERK, and NRF2/ITGB7/FAK signaling pathways [55, 70, 78]; (3) TRIM2 regulates tumor occurrence and development as a downstream target of miR-145, the NR2F1-AS1/miR-493-5p axis, and the hsa-circ-0002286/has-mir-222-5p axis [49, 63, 93]; and (4) TRIM2 participates in the degradation of AXL and interacts with proteins such as SOX10, Snail1, and YAP to regulate tumor progression (Figure 4) [48, 69, 88, 90].

TRIM2 plays a role in regulating tumor progression and is related to various signaling pathways, proteins, and miRNAs. Studies have shown that TRIM2 can be defined as a potential biomarker to evaluate tumor for diagnostic and prognostic evaluation in cancers. TRIM2 promotes tumor growth and metastasis by promoting angiogenesis and regulating the immune microenvironment or inhibiting tumor growth. Regarding the different biological effects of TRIM2 in tumors, in combination with consulting the relevant literature, we proposed the following conjectures and viewpoints that may need further study. (1) There is a relationship between TRIM2 and Bim in disease development, as these proteins may jointly mediate endoplasmic reticulum (ER) stress to regulate tumor progression. In a study of osteosarcoma, after TRIM2 was silenced, DDIT3 was significantly upregulated [55]. DDIT3, the name of the gene encoding C/EBP homologous protein (CHOP, also called GADD153), is the key initiator of ER stress-induced apoptosis; it regulates the expression of p53 upregulated modulator of apoptosis (PUMA) and Bim simultaneously in response to ER stress [100]. Previous studies demonstrated that activation of ERK1/2 signaling initiates the ubiquitination of Bim and its subsequent proteasomal degradation [101] and that TRIM2 expression is induced at the transcriptional level by transcription factors such as CHOP [102]. Several studies on TRIM2 have confirmed the relationship between TRIM2 and Bim. Thus, we speculated that TRIM2 may also ubiquitinate Bim and activate the ER stress response, which may play a role in promoting tumor progression or regulating tumor autophagy and become a potential therapeutic target in cancer. (2) As an oncogenic factor, TRIM2 leads to the production of a large amount of ROS in the tumor microenvironment and promotes tumor progression. In a previous study, TRIM2 was found to accelerate pancreatic cancer progression through the ROS-related NRF2/ITGB7/FAK axis [78], and excessive production of ROS has been considered to be the main mechanism of DMBA-mediated oral carcinogenesis [96]. Previous studies have confirmed that oxidative stress-mediated DNA damage is a critical pathological process during the genesis of various cancers, such as oral cancer, and that instability of the oxidant-antioxidant system can lead to different kinds of pathological diseases, including cancers [103, 104]. Thus, whether TRIM2 mediates oxidative stress and leads to the production of a large amount of ROS in other cancers remains to be further studied. (3) TRIM2 and other TRIM proteins participate in the regulation of cell growth and cell cycle transitions, as previously reported [105]. TRIM2 also plays a role in cell cycle regulation in both pancreatic cancer and ccRCC [78, 92]. Therefore, research on cell cycle regulation by TRIM2, which may provide new insights for the treatment of tumors, needs further study. (4) The interaction between TRIM2 and YAP can regulate the occurrence and development of tumors. Numerous studies have shown that the main roles of YAP are in promoting tumor proliferation, migration, and invasion and that YAP is highly expressed in cancers such as pancreatic cancer and prostate cancer [106, 107]. However, it has been reported that 63% of invasive ductal breast cancers have low expression of YAP [108], and the mechanism by which YAP promotes apoptosis may involve its interaction with the tumor suppressor p73 to enhance apoptosis under conditions of DNA damage [109]. In the study of TRIM2 and CRC, TRIM2 expression has been reported to be negatively correlated with YAP signaling, while TRIM2 also acts as an oncogene in most tumors. The interaction between TRIM2 and Yap thus needs further investigation. (5) TRIM2 participates in the regulation of tumor EMT. In the abovementioned TRIM2 study, TRIM2 was confirmed to regulate the metastasis of CRC through EMT and to regulate the ubiquitination of Snail1 [88, 90]. Snail1 is a key factor in the regulation of EMT, which not only participates in the development of the embryonic mesoderm and the neural tube but also plays an important role in tumor metastasis [110]. Therefore, in-depth research on the involvement of TRIM2 in EMT is worthwhile, which will be helpful for tumor diagnosis, treatment, and prognosis.

## 5. Conclusion

The ability of the TRIM2 protein to antagonize or synergize with other proteins or upstream genes, as well as the related signaling pathways, deserves further study, including determining the roles of TRIM2 in neuroprotection and antiviral therapy. However, TRIM2 is not the only TRIM protein that plays a regulatory role in tumor cells. TRIM2 has not been studied in many tumors, and the mechanism of TRIM2 in tumors is incompletely elucidated. TRIM2 may be a new biomarker or therapeutic target that can be used as an indicator for disease diagnosis, treatment, and prognosis, an important direction for future research.

## Figures and Tables

**Figure 1:** (a) Functional domains of TRIM2 [10]. (b) The 3D structure of TRIM2: cyan: *β*-strand; green: turn; red: *α*-helix (the PDB data were downloaded from https://www.rcsb.org/structure/7B2R).

**Figure 2:** The role of TRIM2 in noncancer diseases and TRIM2-related genes and signaling pathways.

**Figure 3:** Analysis of the differential expression of TRIM2 in tumor tissues and normal tissues based on the TCGA and GTEX databases. Yellow indicates tumor tissue, and blue indicates normal tissue. ∗: *P* < 0.05; ∗∗: *P* < 0.01; ∗∗∗: *P* < 0.001; ∗∗∗∗: *P* < 0.0001. Abbreviations: ACC: adrenocortical carcinoma; BLCA: bladder urothelial carcinoma; BRCA: breast invasive carcinoma; CESC: cervical squamous cell carcinoma and endocervical adenocarcinoma; CHOL: cholangiocarcinoma; COAD: colon adenocarcinoma; DLBC: diffuse large B cell lymphoma; ESCA: esophageal carcinoma; GBM: glioblastoma multiforme; HNSC: head and neck squamous cell carcinoma; KICH: kidney chromophobe; KIRC: kidney renal clear cell carcinoma; KIRP: kidney renal papillary cell carcinoma; LAML: acute myeloid leukemia; LGG: brain lower-grade glioma; LIHC: liver hepatocellular carcinoma; LUAD: lung adenocarcinoma; LUSC: lung squamous cell carcinoma; MESO: mesothelioma; OV: ovarian serous cystadenocarcinoma; PAAD: pancreatic adenocarcinoma; PCPG: pheochromocytoma and paraganglioma; PRAD: prostate adenocarcinoma; READ: rectum adenocarcinoma; SARC: sarcoma; SKCM: skin cutaneous melanoma; STAD: stomach adenocarcinoma; TGCT: testicular germ cell tumors; THCA: thyroid carcinoma; THYM: thymic carcinoma; UCEC: uterine corpus endometrial carcinoma; UCS: uterine carcinosarcoma; UVM: uveal melanoma.

**Figure 4:** Expression and molecular mechanism of TRIM2 in different human cancers. The red ovals represent upregulation of TRIM2 in tumor cells, the green ovals represent downregulation of TRIM2, and the yellow oval represents a lack of differential TRIM2 expression.

**Table 1:** Expression and clinical significance of TRIM2 in various cancers.

Cancer type	Expression	Related gene, protein, and pathway	Mechanism and clinical significance	References
Ovarian cancer	Upregulated	AXL, miR-145, Bim	TRIM2 promotes tumor proliferation and invasion by mediating ubiquitination-mediated degradation of Bim. TRIM2 regulates tumor development by mediating p85*β* to regulate autophagic degradation of AXL.	[48, 49]
Cervical cancer	NS	/	/	[51]
Osteosarcoma	Upregulated	CHOP, PI3K/AKT	TRIM2 regulates the progression and metastasis of osteosarcoma through the PI3K/AKT signaling pathway.	[55]
Neuroblastoma	Upregulated	NR2F1-AS1/miR-493-5p	TRIM2 regulates the progression of neuroblastoma and promotes proliferation and invasion through the NR2F1-AS1/miR-493-5p/TRIM2 axis.	[63]
Breast cancer	Upregulated	SOX10, GPER-MAPK/ERK	The GPER-MAPK/ERK signaling pathway regulates the level of TRIM2, leading to ubiquitination-mediated degradation of Bim, which promotes tumor proliferation and invasion and promotes tumor cell resistance to tamoxifen.	[69, 70]
Follicular thyroid carcinoma	Downregulated	/	TRIM2 exhibits higher expression in noninvasive FTC than in invasive FTC; the classification of FTC can be further refined and can be used to guide treatment and assess prognosis.	[75]
Pancreatic cancer	Upregulated	NRF2/ITGB7/FAK	TRIM2 promotes tumor proliferation, invasion, and metastasis through ROS-related NRF2/ITGB7/FAK axis activity and participates in cell cycle regulation.	[78]
Melanoma	Upregulated	/	TRIM2 overexpression is associated with poor prognosis and promotes tumor proliferation and invasion.	[83]
Lung adenocarcinoma	Upregulated	Snail1	TRIM2 promotes the proliferation, invasion, and migration of lung cancer cells by regulating the ubiquitination-mediated degradation of Snail1 and regulates EMT in cooperation with Snail1.	[88]
Colorectal cancer	Upregulated	YAP	TRIM2 overexpression could promote the proliferation and invasion of CRC cells, the expression of TRIM2 correlated with tumor stage and age, and TRIM2 was negatively correlated with YAP.	[90]
Clear cell renal cell carcinoma	Downregulated	hsa-circ-0002286/has-mir-222-5p	Lower TRIM2 expression is associated with the G2/M checkpoint, EMT, hypoxia pathway, and Myc signaling pathway; TRIM2 expression is correlated with tumor recurrence, OS, and TNM stage.	[92, 93]
Oral buccal mucosa cancer	Downregulated	/	TRIM2 may provide insight for the treatment and chemoprevention of buccal mucosa cancer.	[96]

## Data Availability

The data used to support the findings of this study are included within the article.
